# Video Analysis in Sports by Lightweight Object Detection Network under the Background of Sports Industry Development

**DOI:** 10.1155/2022/3844770

**Published:** 2022-08-21

**Authors:** Yifei Zheng, Hongling Zhang

**Affiliations:** ^1^Physical Department, Chang'an University, Xi'an 710064, Shaanxi, China; ^2^Physical Institute, Yan'an University, Yan'an 716000, Shaanxi, China

## Abstract

This study uses the video image information in sports video image analysis to realize scientific sports training. In recent years, game video image analysis has referenced athletes' sports training. The sports video analysis is a widely used and effective method. First, the you only look once (YOLO) method is explored in lightweight object detection. Second, a sports motion analysis system based on the YOLO-OSA (you only look once-one-shot aggregation) target detection network is built based on the dense convolutional network (DenseNet) target detection network established by the one-shot aggregation (OSA) connection. Finally, object detection evaluation principles are used to analyze network performance and object detection in sports video. The results show that the more obvious the target feature, the larger the size, and the more motion information contained in the sports category feature, the more obvious the effect of the detected target. The higher the resolution of the sports video image, the higher the model detection accuracy of the YOLO-OSA target detection network, and the richer the visual video information. In sports video analysis, video images of the appropriate resolution are fed into the system. The YOLO-OSA network achieved 21.70% precision and 54.90% recall. In general, the YOLO-OSA network has certain pertinence for sports video image analysis, and it improves the detection speed of video analysis. The research and analysis of video in sports under the lightweight target detection network have certain reference significance.

## 1. Introduction

With the continuous maturity of “Internet +” technology, the sports industry has gradually developed in the direction of wisdom, inclusiveness, and services. Smart technology is used to collect and distinguish the needs of mass sports accurately. The concept of sharing integrates sports resources and realizes the online and offline integration of the sports industry by enriching sports service projects and innovating development concepts. Based on meeting the needs of mass sports, it realizes the multiple values of the sports industry [1–3]. With the help of social media, the public has become an important force in promoting the high-quality development of the sports industry. The public uses pedometer applications (APP) and social media platforms to share and exchange sports experiences. This behavior has formed a new sports social model, helping sports become a way of life for the public to share and communicate [4, 5]. However, when videos in sports are analyzed, there are certain drawbacks. Most sports videos require the experience of professional scouts [6]. With the gradual penetration of intelligent video analysis applications in various industries, from sports to climate science, intelligent video analysis applications in various industries are changing the future [7]. Intelligent video analytics is also known as visual artificial intelligence (AI), or visual AI for short. This technology can turn complex video data into actionable insights to help humans manage urban traffic, improve urban planning, increase safety in public spaces, and even curate theatrical performance content [8, 9]. Visual AI can improve the operational efficiency of sports venues, improve the quality of live streaming, and evaluate athlete performance for athletes and fans of the sports world. It also allows users to exercise at home to adjust their workouts under the guidance of a fitness trainer [10].

The Swiss “Dartfish” is the most advanced and widely used professional motion video analysis system in the world. It is powerful and comprehensive, with professional, project tactical analysis, training, and other functions, especially multiscreen comparison, video overlap analysis, key action decomposition, video marking, and other functions, which is particularly suitable for the sports field [11]. Therefore, Dartfish not only uses diagrams for analysis and time stamping but also enables real-time actions to be compared with typical characteristics, allowing experts and athletes to see the most important elements immediately [12]. Bilai and Hanif used histogram of oriented gradient (HOG) for feature extraction and support vector machine (SVM) as a classifier for pedestrian detection. After extensive testing, HOG hybrid SVM is a pedestrian detection method with a better balance between speed and effect [13]. In 2019, fully convolutional one-stage object detection (FCOS) in object detection algorithms prevailed in the society. The algorithm uses detection heads with shared weights, that is, using the same set of convolutions to predict detection boxes for the multiscale feature map of feature pyramid network (FPN). Then, each layer uses a learnable scale value to solve the object detection problem in a pixel-by-pixel prediction manner, like semantic segmentation [14]. The FCOS algorithm is not the first to propose the use of a full-scroller network for object detection. DenseBox is also an algorithm based on fully convolutional network (FCN) [15]. FCOS will predict a 4-dimensional vector plus a piece of category information for each point on the feature map, that is, each point on the feature map of width by height (*W* × *H*). Channels are set to 5. In fact, this is like semantic segmentation, except that there is four more bounding box offset information [16]. When FCOS is lightweight, the model effect is not as good as expected because the centerness branch of FCOS is difficult to converge on lightweight models [17]. Chen and Qin proposed the generalized focal loss function. This function can remove the centerness branch of FCOS and save a lot of convolutions on this branch, thereby reducing the computational overhead of the detection head, which is very suitable for lightweight deployment on mobile terminals [18]. Koo et al. used you only look once (YOLO) to achieve real-time object detection used in cutting-edge technologies such as self-driving cars [19].

Target detection and recognition methods based on deep learning have become mainstream. The study deeply discusses the regression-based target detection and recognition algorithm and optimizes the YOLO method. The lightweight target detection method is applied to sports, which not only combines the current technical methods with practice but also highlights the characteristics of the era of sports operation. These provide a video analysis research method for sports and a new path for the economic development of the sports industry.

This study aims to use the video image information in sports video image analysis to realize scientific sports training. First, the YOLO method in lightweight object detection is explored. Second, based on the one-shot aggregation (OSA) connection, the dense convolutional network (DenseNet) is established, and the sports analysis system is established based on the you only look once-one-shot aggregation (YOLO-OSA) target detection network. Finally, object detection evaluation principles are used to analyze network performance and object detection in sports video. This study has certain reference significance for the research and analysis of video in sports under the lightweight target detection network.

## 2. Object Detection Network Method

### 2.1. YOLO Target Detection

Deep learning target detection has been developed for many years, from two-stage to one-stage, from anchor-base to anchor-free, and then to a transformer for target detection. Various methods are blooming. However, in mobile target detection algorithms, anchor-base models such as the YOLO series and single shot multiBox detector (SSD) have always dominated [20]. YOLO can input a picture and directly output the result, including the name and score of the box and objects in the box [21]. The principle of YOLO target detection is shown in Figure 1.

In Figure 1, first, the size of the sports picture is fixed. The input image is divided into an *n∗n* grid, and classification and localization are performed on each grid. Compared to sliding windows, this greatly reduces the amount of computation. Before YOLO performs detection, the image has meshed. When an object's center falls within a grid, that grid is responsible for predicting the object. Each grid needs to predict a bounding box, and each bounding box needs to predict a confidence value in addition to its own position. This confidence value represents the confidence of the object in the predicted box (what object is contained in the grid and the accuracy of predicting this object) and the multiple information predicted by this box. By dividing the image into multiple blocks, a tensor with the same number of blocks is directly output. The prediction vector of each block determines whether it has a target and what type it is, and the correct calculation of the specific position is shown in the following equation:

(1) $$\begin{array}{c} \mathrm{Pr}\left(\text{Object}\right)*IOU_{\text{pred}}^{\text{truth}}. \end{array}$$

In the equation, if an object falls in a grid unit, then the first item takes 1; otherwise, it takes 0. The second term is the intersection over union (IoU) value between the predicted bounding box and the actual bounding box. When there is no object in the box, the entire confidence will become 0. However, with the evolution of time, there is a lack of lightness in the application, and the practical application is not strong.

### 2.2. Lightweight Object Detection Network Based on OSA Connection

Different networks are introduced to optimize the object detection model. The inception series is different from the residual network (ResNet). The inception network mainly improves the network structure from the width of the network to improve the expressive ability of the network. ResNet mainly improves the network structure from the depth of the network to improve the expressive ability. DenseNet explores the potential of the network through feature map reuse. DenseNet can make the input of each layer of the network become the superposition of all previous layers. Then, its feature map is passed to all subsequent network layers [22]. The 5-layer dense block structure of the DenseNet network with a growth rate of 4 is shown in Figure 2.

In Figure 2, a growth rate of 4 means that the output feature map dimension of each dense layer is 4. A 5-layer dense block represents 5 BN-ReLU-Conv (3*∗*3) layers. All layers are directly connected to ensure the maximum information flow between layers. In order to maintain the feed-forward feature, the input of each layer is the output of all previous layers, and its own feature map results are also used as the input of the subsequent layers. DenseNet consists of dense blocks. In these blocks, the layers are closely connected, and each layer takes its input from the output feature map of the previous layer. This extreme reusability of residuals results in deep supervision, with each layer receiving more supervision from the previous layer, so the loss function will react accordingly. In dense blocks, a single block consists of batch normalization, ReLU activation, and 3 × 3 convolution. *Transition Layer*. In ResNet, the summation of residuals is performed, while DenseNet concatenates all feature maps together. Batch normalization, convolutional layer, and average pooling constitute the transition layer. DenseNet's convolutions generate fewer feature maps. DenseNet has lower requirements for wide layers. With tight connections between layers, it learns features with little redundancy. The number of output feature maps of a layer is defined as the growth rate. Ultimately, the growth rate controls how much new information each layer contributes to the global [23]. The input and output transformation graphs of the first convolutional layer in the dense block are shown in the following equation:

(2) $$\begin{array}{c} x_{l}=H_{l}\left(\left[x_{0},x_{1,\ldots ,x_{l-1}}\right]\right). \end{array}$$

In the equation, [*x*_0_, *x*_1,…,*x*_*l*−1__] is the output feature of the 0th layer to the *l* − 1th layer in the module. *H*_*l*_ completes nonlinear transformation for the *l*th convolutional layer. The residual connection module of the input and output transformation of the first convolutional layer is shown in the following equation:

(3) $$\begin{array}{c} x_{l}=H_{l}\left(x_{l-1}\right)+x_{l-1}. \end{array}$$

In the equation, *l* is the representation layer, *x*_*l*_ is the output of the *l* layer, *x*_*l*−1_ is the output of the *l* − 1 layer, and *H*_*l*_ is a nonlinear transformation. Therefore, for ResNet, the output of layer *l* is the output of layer *l* − 1 plus a nonlinear transformation of the output of layer *l* − 1. The core module of DenseNet is the dense block. This dense connection aggregates all previous layers, resulting in a linear increase in the input of each layer. The output of each layer is fixed size, limited by floating-point operands and model parameters. The problem with it is that the input and output are inconsistent. Currently, the network model is not optimal. In addition, due to the large input, DenseNet uses a 1 × 1 convolutional layer to compress the features first. The introduction of this extra layer is detrimental to the efficient computation of the graphics processing unit (GPU). Therefore, although DenseNet's floating-point operations and model parameters are not large, the inference is not efficient. When the input is large, more memory and inference time are often required. Therefore, although the floating point operations (FLOPs) and model parameters of DenseNet are not large, the inference is not efficient. It tends to require more memory and inference time when the input is larger. The OSA connection is proposed, as shown in Figure 3.

In Figure 3, *F* is a floating-point operand. *X* is the output value of all layers. That is, all previous layers are aggregated only at the last time. This connection change will solve the problems described earlier in DenseNet. The number of input channels of each layer is fixed, assuming that the number of output channels is consistent with the input to obtain the smallest memory access cost and no longer needs 1 × 1 convolutional layers to compress features. The OSA module is computationally efficient [24]. The OSA module is shown in Figure 4.

In Figure 4, the module contains *m* convolutional layers. *f* is the output of each convolutional layer along with the input channel. *g* is the channel number of the input module. At the end of the OSA module, the outputs of the *m* convolutional layers are superimposed with the input channels of the OSA module. If the number of superimposed is too large, a 1*∗*1 convolutional layer is added at the end of the OSA module for the compression module. Finally, each stage uses a max-pooling layer for downsampling. Like other networks, the number of feature channels is increased after each downsampling.

### 2.3. Sports Video Analysis System

Sports is a social activity, in which people follow the growth and development laws of the human body and the laws of physical activity through physical exercise, technology, training, competitive competitions, and other methods to enhance physical fitness, improve the level of sports technology, and enrich cultural life. It is a general term for all competitive physical activities that provide entertainment to participants through the use, maintenance, or improvement of physical fitness, and organized or unorganized participation. There are hundreds of sports in the world, and their forms vary widely. Some only require two people to complete, while others require multiple teams to complete [25]. The main categories of sports are listed in Table 1.

In Table 1, different sports models have the characteristics of fast target movement and fast change of target speed in sports videos. Therefore, four motion models such as uniform velocity, uniform acceleration, rest, and collision are proposed. In sports events, single data statistics and unstructured video recordings have certain limitations and do not produce much value. Combining statistics and video to structure and refine video data can assist sports events and sports training and provide valuable solutions. The 3D panoramic video surveillance and video processing flow are shown in Figure 5.

In Figure 5, the video image is preprocessed and noise removed. The geometrically distorted images are corrected. Additionally, a histogram equalization image enhancement algorithm is incorporated. The images with lower definition are image enhanced, and the frame image registration algorithm is used to complete the image feature point detection, feature description, and feature matching. The overlapping parts between the images are aligned. The image to be stitched is transformed into the coordinate system of the reference image to form a complete image. The frame image fusion algorithm is used to fuse the overlapping areas of the splicing so that the color gradually transitions, ensures the smooth transition of the splicing boundary, eliminates the splicing line, and generates a smooth and seamless panoramic video image. Multiple monitoring probes are equipped with an embedded processor, a video acquisition module connected with the embedded processor for video image acquisition in the monitoring area, and a video processing module for video processing of the collected video images and positioning of the probe position [26]. In addition, for moving video, the principle diagram of the background difference method in the process of target detection is shown in Figure 6.

In Figure 6, the basic idea of the background difference method is to compare the input image with the background model. The moving objects are segmented by judging changes in features such as grayscale or using changes in statistical information such as histograms. First, the background image frame B and the stored background image are established [27]. The difference in image calculation is shown in the following equation:

(4) $$\begin{array}{c} D_{n}\left(x,y\right)=\left|f_{n}\left(x,y\right)-B\left(x,y\right)\right|, \end{array}$$

where *B*(*x*, *y*) and *f*_*n*_(*x*, *y*) are the grayscale values of the pixels corresponding to the background frame and the current frame. *D*_*n*_(*x*, *y*) is the grayscale value of the differential image. The binarization processing calculation is shown in the following equation:

(5) $$\begin{array}{c} R_{n}^{\prime }\left(x,y\right)=\left\{\begin{array}{cc} 255, & D_{n}\left(x,y\right)>1,\\ 0, & \text{else}. \end{array}\right. \end{array}$$

In the equation, *R*_*n*_′(*x*, *y*) is a binarized image, in which the point with a gray value of 255 is the foreground (moving target) point, and the point with a gray value of 0 is the background point. When the subtraction of the current frame and the background image is greater than a certain threshold, the pixel is determined to be the foreground target: the input image is subtracted from the background image, and *T* is the threshold or difference. After thresholding, the point corresponding to the 0 value in the image is the background image, and the point corresponding to the 1 value is the moving pixel in the scene. The sports analysis system based on the YOLO-OSA target detection network is shown in Figure 7.

In Figure 7, target detection in sports videos is solved based on the YOLO-OSA target detection network. First, the video obtained through the camera is punched. Second, the target detection network enters the working mode to perform sports video control, target calibration, target tracking, and motion tracking analysis.

### 2.4. Principles of Model Evaluation

The IOU of the standard frame predicted by the system model and the real frame is greater than or equal to 0.5, and the sports target recognition is correct. The system adopts the accuracy rate, precision rate, recall rate, and average precision as the system evaluation principles [28]:

(1) The accuracy rate is the percentage of correctly predicted samples in the total samples. Although the accuracy rate can judge the correct overall rate, in the case of unbalanced positive and negative samples, the evaluation index of the accuracy rate has a great defect. For example, in the total sample, positive samples account for 90%, and negative samples account for 10%. In this case, it is only necessary to predict all samples as positive samples to get high accuracy of 90%. The calculation is shown in the following equation:
  (6) $$\begin{array}{c} A\left(\text{accuracy}\right)=\frac{\text{TP}+\text{TN}}{\text{TP}+\text{TN}+\text{FP}+\text{FN}}. \end{array}$$
True positive (TP) is the number of positive samples that are correctly identified. True negative (TN) is the number of correctly identified negative samples. False positive (FP) is the number of negative samples that are incorrectly identified as positive samples. False negative (FN) is the number of positive samples that are falsely identified as negative samples.
(2) *Accuracy Rate*. The accuracy rate is also called the precision rate. The percentage of positive samples that are correctly predicted to all detected (predicted as positive) samples is for the prediction results. The calculation is shown in equation (7):
  (7) $$\begin{array}{c} P\left(\text{precision}\right)=\frac{\text{TP}}{\text{TP}+\text{FP}}. \end{array}$$
(3) *Recall Rate*. The recall rate is the proportion of positive samples that are correctly predicted to all positive samples (ground truth). It is for the original sample. The calculation is shown in the following equation:
  (8) $$\begin{array}{c} R\left(\text{recall}\right)=\frac{\text{TP}}{\text{TP}+\text{FN}}. \end{array}$$
(4) *Average Precision*. Average precision is a performance metric for this class of algorithms that predict target locations as well as classes. The calculation is shown in the following equation:
  (9) $$\begin{array}{c} AP\left(\text{average precision}\right)=\frac{\sum_{0,0.1,\ldots ,1.0}P_{\text{smooth}}\left(i\right)}{11}. \end{array}$$

In the equation, *P* is the value of different recall rates. ∑_0,0.1,…,1.0_*P*_smooth_(*i*) is the precision of the recall rate, Recall = {0,0.1, 0.2, 0.3, 0.4, 0.5, 0.6, 0.7, 0.8, 0.9, 1}. Mean average precision (MAP) is the average of multiple categories of AP. Mean means that the AP obtained under each category is averaged. The value range of MAP is [0, 1]. In this range, the larger the MAP value, the higher the average accuracy.

## 3. Results and Discussion

### 3.1. Analysis of Sports Video Target Detection under the YOLO-OSA Target Detection Network

Through the sports video analysis under different sports types under the YOLO-OSA target detection network, the sports video target detection analysis is shown in Figure 8.

Figure 8 shows the detection accuracy of video objects in each category of sports by YOLO-OSA. The target detection accuracy rate of competitive sports is 61.30%, the recall rate is 66.80%, and the MAP value is 62.50%. The accuracy rate of entertainment sports and target detection is 23.30%, the recall rate is 45.50%, and the MAP value is 36.30%. The accuracy rate of mass sports target detection is 21.70%, the recall rate is 54.90%, and the MAP value is 39.40%. The accuracy rate of medical sports target detection is 18.30%, the recall rate is 55.90%, and the MAP value is 35.70%. According to the sports category characteristics, the more obvious the target features, the larger the size, and the more motion information contained, the more obvious the effect of the detected target.

### 3.2. The Influence of Different Sports Video Input Resolutions on the YOLO-OSA Target Detection Network

Sports video images at different resolutions test the performance of the YOLO-OSA object detection network. The “horizontal pixel number*∗*vertical pixel number” of the video image is used to express the video image, and the videos with different pixel sizes of 416*∗*416, 608*∗*608, and 832*∗*832 are detected, respectively. The influence of sports video images at different resolutions on the YOLO-OSA target detection network is shown in Figure 9.

In Figure 9, the higher the resolution of the sports video image, the higher the model detection accuracy of the YOLO-OSA target detection network, and the richer the visual video information. However, the higher the resolution of the sports video image, the longer the detection time of a single frame, which means the higher the resolution of the video image. The amount of computation and access to the network reduces the computation speed of the network. Therefore, in sports video analysis, video images of appropriate resolution size are selected for input into the system.

### 3.3. Performance Comparison of Sports Video Analysis under Different Networks

The core idea of YOLO is to use the entire image as the network's input. Multiple downsampling layers are employed at the output layer to regress the location of the bounding box and the class, to which it belongs. The object features learned by the network are not fine, so it also affects the detection effect. The OSA connection and the digital signal processing (DSP) method are used to make up for the shortcomings of the YOLO method. Each stage of the OSA connection uses a max-pooling layer for downsampling and no longer requires a 1 × 1 convolutional layer to compress features. Therefore, the OSA module is GPU computationally efficient. You only look once-digital signal processing (YOLO-DSP) algorithm is feasible in identifying medium or large-size objects in unrestricted natural scenes. The proposed lightweight target detection network uses the YOLO network, YOLO-OSA network, and you only look once-digital signal processing (YOLO-DSP) network for performance analysis under the sports video dataset. A dataset is obtained from the University of Florida Sports Behavior Database, which consists of a series of actions collected from various sports, containing 150 sequences. The resolution is 720*∗*480, and this set represents the natural action pool in various scenes and viewpoints. The resolution is uniformly set to 800, and the confidence is set to 0.01. The performance comparison of sports video analysis under different models is shown in Figure 10.

In Figure 10, the network structure and the multiscale improved YOLO-OSA network obtained 21.70% precision and 54.90% recall. This is an increase of 6.80% and 6.50%, respectively, compared to YOLO. The YOLO-DSP network achieves 13.20% precision and 43.90% recall. The average detection accuracy of the YOLO-OSA network is higher than other networks and 10.00% higher than that of the YOLO-DSP, indicating that the YOLO-OSA network has a certain pertinence for the analysis of sports video images and improves the detection speed.

## 4. Conclusions

At present, most of the target tracking methods are based on a static background. The frame difference between the target and the background is used to extract the contour information of the moving target to obtain the moving position of the target. However, in sports videos, the camera often moves violently, and the background changes every moment, so it is difficult to use the background frame difference to obtain the moving position of the target. Through the YOLO-OSA target detection network to conduct sports video analysis research, the results show that the average detection accuracy of the YOLO-OSA network is higher than that of other networks. Sports video image analysis has certain pertinence and improves the detection speed. Under the lightweight target detection network, video research and analysis in sports have certain reference significance. The development of the sports industry itself is very important for national economic development. In the future, the sports industry can use scientific definitions and suggestions in sports video analysis to make standardized and creative sports industry development. This industry will be able to regulate the marketization of the sports industry better, thus promoting the development of the national social economy. In terms of the design model method, this study is based on the YOLO implementation model. In view of the endless network structures of efficient feature extraction of lightweight target detection networks, it is hoped to improve the detection accuracy of the lightweight target while ensuring the detection speed. In sports videos, the increase in data amount reduces the processing speed. In the future, the study will be able to design a more efficient detection model for unified training of different targets.

## Figures and Tables

**Figure 1:** The principle of YOLO target detection.

**Figure 2:** DenseNet 5-layer dense block structure with a net growth rate of 4.

**Figure 3:** OSA connection.

**Figure 4:** OSA module.

**Figure 5:** 3D panoramic video surveillance and video processing flow.

**Figure 6:** Schematic diagram of background difference method.

**Figure 7:** Sports analysis system based on YOLO-OSA target detection network.

**Figure 8:** Sports video target detection analysis.

**Figure 9:** Influence of sports video images at different resolutions on the YOLO-OSA target detection network.

**Figure 10:** Performance comparison of sports video analysis under different networks.

**Table 1:** Main categories of sports.

Sports category	Features
Athletics	Adversarial, mobilizing, technical, international, and recognized
Entertainment sports	Amateur, recreational, and recreational
Popular sports	Extensive
Medical sports	Active, restorative, and therapeutic

## Data Availability

The data used to support the findings of this study are included within the article.
